# The Compatibility of Alisma and Atractylodes Affects the Biological Behaviours of VSMCs by Inhibiting the miR-128-5p/p21 Gene

**DOI:** 10.1155/2022/7617258

**Published:** 2022-07-07

**Authors:** Wei Wei, Yang Jie Zhou, Ju Lian Shen, Lu Lu, Xin Ru Lv, Tao Tao Lu, Pei Tao Xu, Xie Hua Xue

**Affiliations:** ^1^The Affiliated Rehabilitation Hospital, Fujian University of Traditional Chinese Medicine, Fuzhou, China; ^2^College of Rehabilitation Medicine, Fujian University of Traditional Chinese Medicine, Fuzhou, China; ^3^Fujian Provincial Rehabilitation Industrial Institution, Fujian Provincial Key Laboratory of Rehabilitation Technology, Fujian Provincial Key Laboratory of Cognitive Rehabilitation, Fuzhou, China

## Abstract

**Objective:**

The compatibility of Alisma and Atractylodes (AA) has been estimated to exhibit antiatherosclerotic effects, but the mechanism remains unclear. This study aimed to identify the role of AA in oxidized low-density lipoprotein (ox-LDL)-induced vascular smooth muscle cell (VSMC) behaviours and to explore the effects of microRNAs (miRNAs).

**Methods:**

A scratch wound-healing assay was used to detect the migration of VSMCs, and immunocytochemistry and western blotting for SM22ɑ were used to evaluate phenotypic transformation. Bromodeoxyuridine (BrdU) immunocytochemistry and flow cytometry were applied to detect the proliferation of VSMCs. miRNA microarray profiling was performed using Lianchuan biological small RNA sequencing analysis. VSMCs were transfected with the miR-128-5p mimic and inhibitor, and the migration, phenotypic modulation, and proliferation of VSMCs were investigated. The 3′UTR-binding sequence site of miR-128-5p on the p21 gene was predicted and assessed by luciferase assays.

**Result:**

AA and the extracellular regulated protein kinase 1/2 (ERK1/2) blocker U0126 markedly inhibited migration, elevated smooth muscle 22*α* (SM22*α*) expression, repressed VSMC proliferation, elevated miR-466f-3p and miR-425-3p expression, and suppressed miR-27a-5p and miR-128-5p expression in ox-LDL-induced VSMCs. miR-128-5p targets the tissue inhibitor of metalloproteinases (TIMPs), silent information regulator 2 (SIRT2), peroxisome proliferator-activated receptor (PPAR), and p21 genes, which are linked to the behaviours of VSMCs. The miR-128-5p mimic promoted the migration and proliferation of VSMCs and suppressed p21, p27, and SM22ɑ expression. The inhibitor increased p21, p27, and SM22ɑ expression and repressed the migration, phenotypic transformation, and proliferation of VSMCs. miR-128-5p directly targeted the 3′UTR-binding sequences of the p21 gene, negatively regulated p21 expression, and supported the proliferation of VSMCs.

**Conclusion:**

Our research showed that the migration, phenotypic transformation, and proliferation of ox-LDL-induced VSMCs were repressed by AA through inhibiting miR-128-5p by targeting the p21 gene, which may provide an effective option for the treatment of atherosclerosis.

## 1. Introduction

Atherosclerosis (AS), the main pathological process of arterial lesions, is the cause of the majority of cardiovascular and cerebrovascular diseases. It has been shown that inflammation caused by oxidized low-density lipoprotein (ox-LDL) contributes to the occurrence and development of AS [1], which can promote vascular smooth muscle cell (VSMC) migration, proliferation, and transformation from a contractile to a synthetic phenotype [2–6]. A large number of cytokines, extracellular matrix (ECM), and matrix metalloproteinases (MMPs) are synthesized and secreted by synthetic VSMCs during the progression of AS [7, 8]. The migration, phenotypic transformation, and proliferation of VSMCs lead to vascular wall remodeling, which is mediated by activation of extracellular regulated protein kinases 1/2 (ERK1/2) signalling [9].

MicroRNAs (miRNAs) are small noncoding sequences involved in the negative regulation of gene expression. A series of cellular pathophysiological mechanisms involved in AS (e.g., differentiation, proliferation, and signalling pathways) are under the control of miRNAs. miRNAs are recognized as important regulators of lipid metabolism, inflammatory mediators, and VSMC behaviours in the progression of AS [10]. Several studies have shown that miRNAs play multiple roles in the phenotypic transformation, migration, and proliferation of VSMCs by inhibiting ERK1/2 activation [11, 12], partly by regulating the tissue inhibitor of metalloproteinases (TIMPs)-MMPs and p21-cyclins interactions [13–18].

Alisma and Atractylodes (AA) is a classic traditional Chinese medicinal formula that first appeared in the “Synopsis of Prescriptions of the Golden Chamber.” AA exhibits multiple pharmacological actions [19–22]. It has been reported that Alisma orientale has a protective effect on acute lung injury through an anti-inflammatory effect by repressing the NF-kappa B pathway [20]. The extract of Alisma orientale exerted a protective effect on nonalcoholic fatty liver disease and palmitate-induced cellular injury [21, 22], suggesting that it could be a potential treatment for abnormal lipid metabolism syndrome. Several studies have shown that AA represses lipid deposition in macrophage-derived foam cells [23]. Alisol A 24-acetate, an active extract derived from Alisma orientale, inhibited migration and repressed the transformation from a contractile to a synthetic phenotype in ox-LDL-treated VSMCs by inhibiting ERK1/2 signalling [9]. However, little is known about the mechanisms of AA on VSMC migration, phenotypic transformation, and proliferation. This study aimed to investigate the impact of AA on ox-LDL-induced VSMCs and explore the underlying mechanisms of miRNAs.

## 2. Materials and Methods

### 2.1. Ethical Statement and Animals

All Sprague Dawley (SD) rats, provided by Fujian University of Traditional Chinese Medicine (Fujian, China), were treated following the Suggested Guidelines for the Care and Use of Laboratory Animals 2006 administered by the Ministry of Science and Technology, China. This study was approved by the Animal Care and Use Committee of the Fujian University of Traditional Chinese Medicine (permission number: 2015–016). All rats were housed in facilities and provided food and water ad libitum.

### 2.2. Preparation of AA-Containing Serum

AA-containing serum was prepared according to a previous study [23]. In brief, the rats were assigned to 2 groups and then given AA and 0.9% NaCl by oral gavage at 4 mL twice daily for 7 d. Then, blood samples were collected from the rat abdominal aorta following induction of anaesthesia with diazepam/ketamine (1 : 1) (1 mL/1000 g), and serum was separated by centrifugation at 3000 r·min^−1^ at 4°C for 10 min. After the bacteria were filtered with a microporous membrane, the serum was inactivated in a 56°C water bath for 30 min and then stored at −20°C for the study.

### 2.3. VSMC Isolation and Culture

VSMCs were prepared from rats as described previously [9]. VSMCs were removed from the rat thoracic aorta and cultivated with Dulbecco's modified Eagle's medium (DMEM)/F12 (GIBCO, Life Technologies, USA) and 20% foetal bovine serum (GIBCO, Life Technologies, USA) containing penicillin and streptomycin solution (1 : 1) (GIBCO, Life Technologies, USA) at 37°C with 5% CO_2_. VSMCs grown to 85%–90% confluence were forced into quiescence by FBS-free serum starvation for 24 h. Then, VSMCs were assigned to four groups. Control group: VSMCs were cultured in DMEM/F12 with 20% normal rat serum; ox-LDL group: VSMCs were cultured with 20% normal rat serum and 50 mg·L-1 ox-LDL (Peking Union-Biology Co, Ltd., Beijing, China); AA group: VSMCs were cultured in DMEM/F12 supplemented with 20% AA and 50 mg·L-1 ox-LDL; and U0126 group: VSMCs were treated with 10 *μ*mol·L-1 U0126 (Sigma-Aldrich, Inc., St. Louis, MO, USA) and 50 mg·L-1 ox-LDL.

### 2.4. VSMC Migration Assay

VSMC migration was assayed by a scratch wound healing assay. Well-functioning VSMCs (1.0 × 105 cells/well) at 60–70% confluence were incubated in a 6-well dish and starved with DMEM/F12 containing 0.5% FBS for 12 h. A linear scratch wound was made at the centre of the cell monolayer with a 200 *µ*L pipette tip and washed twice with PBS. VSMCs in the assigned groups were treated as described above in DMEM/F12 with 20% FBS. Cells were cultured for 24 h at 37°C with 5% CO_2_, and then the images of scratches were observed using a Leica DM IL LED inverted microscope (Wetzlar, Germany) and LAS Interactive Measurement imaging analysis software (Leica Microsystems, Mannheim, Germany).

### 2.5. Detection of Phenotypic Transformation in VSMCs

Immunofluorescence assays were used to detect the expression of the VSMC phenotypic marker smooth muscle 22*α* (SM22*α*). Logarithmic-phase VSMCs (1 × 105 cells/well) were incubated onto a cover glass in 6-well plates. VSMCs in the assigned groups were treated for 24 h as described above. VSMCs were fixed in 4% paraformaldehyde for 15 min, rinsed with PBS, passed through 0.3% Triton X-100 for 15 min, blocked with goat serum for 30 min, cocultured with anti-rabbit SM22*α* monoclonal antibody (1 : 200; Proteintech, USA), rinsed with PBS, incubated with secondary antibody (1 : 200; Proteintech, USA) and DAPI dye solution (100 ng·mL-1, BOSTER Biological Technology, China), drained from the dye solution, and observed under a fluorescence microscope. Five fields of vision were randomly photographed from each well plate and comprehensively analysed using imaging processing software (Image-Pro Plus v6.0, Media Cybernetics, Bethesda, MD, USA).

### 2.6. Secretion of MMP-2 and MMP-9 Detected by ELISA

The secretion of MMP-2 and MMP-9 in VSMCs was detected by ELISA. The cells were treated for 24 h as described above, and the culture supernatants were harvested. According to the manufacturer's instructions, the expression of MMP-9 and MMP-2 was measured in the cell culture supernatant using a Sandwich ELISA kit (BOSTER Biological Technology, China).

### 2.7. VSMC Proliferation Assay

BrdU immunocytochemistry and flow cytometry were used to measure the proliferation of VSMCs. VSMCs (1 × 105 cells/well) were seeded onto 6-well plates and incubated in DMEM/F12 supplemented with 20% FBS for 24 h. Quiescent VSMCs at 60–70% confluence in DMEM/F12 with 0.5% FBS were grouped as described above and cultivated with BrdU (30 *μ*mol/L) for 24 h following the instructions of the FITC-BrdU cell proliferation assay kit (BOSTER Biological Technology, China) and detected by flow cytometry at a 488 nm excitation wavelength and 520 nm emission wavelength. BrdU expression was assessed by immunocytochemical staining following the manufacturer's instructions. Five fields of vision were randomly photographed from each well plate and comprehensively analysed using image-processing software (Image-Pro Plus v 6.0, Media Cybernetics, Bethesda, MD, USA). The positive cells were detected by BrdU manifesting pale-yellow or deep-tan staining, while negative cells exhibited nonspecific background staining.

### 2.8. miRNA Microarray Assay and miRNA Target Gene Interactions

Total RNA was extracted from VSMCs. miRNA microarray profiling was performed using Lianchuan Biological Small RNA Sequencing Analysis (Lianchuan Bio, China) according to the manufacturer's recommended protocol. Small RNA sequencing library preparation was performed using the TruSeq Small RNA Sample Prep Kit (Illumina, San Diego, USA). After the library preparation work was completed, the constructed library was sequenced using Illumina HiSeq 2000/2500, and the sequencing read length was 1 × 50 bp. The potential target genes of miRNAs were searched with the TargetScan 7.2 database and miRDB. The target gene interactions of miRNAs were determined according to the database.

### 2.9. Transfection of VSMCs with miR-128-5p Mimic and Inhibitors

VSMCs were kept completely synchronous with serum starvation for 24 h before transfection. VSMCs (2–3 × 105 cells/well) at 60%–70% confluence were treated for 24 h as described above and transfected with 50 nM miR-128-5p mimic, miR-128-5p inhibitor, mimic-negative control (NC), or inhibitor NC using siRNA-Mate plus (GenePharma, Shanghai, China) according to the manufacturer's protocol. The miR-128-5p mimic, inhibitor, mimic NC, and inhibitor NC were designed and synthesized by GenePharma (Shanghai, China). The sequences were as follows: 5′-UCAGUGCUACGGCCCCGUU-3′ (miR-128-5p mimic); 5′-UUCUCCGAACGUGUCACGUTT-3′ (miR-128-5p mimic NC); 5′-UCUCAGUGCUACGGCCCCG-3′ (miR-128-5p inhibitors); and 5′-CAGUACUUUUGUGUAGUACAA-3′ (miR-128-5p inhibitors NC). Total RNA was isolated from VSMCs after transfection using TRIzol (Invitrogen, Carlsbad, CA, USA) following the manufacturer's manual. miRNA expression was detected by qRT-PCR with a One Step SYBR® PrimeScript™ RT–PCR kit II (Takara, Tokyo, Japan) according to the manufacturer's protocol.

### 2.10. Western Blot Analysis of the Protein Expression of p21, p27, and SM22ɑ

After treatment for 24 h as described, the cells were collected and lysed with RIPA buffer (Tris-HCl: 50 mM (pH 8.0); NP-40 : 1.0%; Na-deoxycholate: 1.0%; NaCl: 150 mM; SDS: 0.1%; and PMSF: 0.05 mM), and the protein concentration was assessed using the BCA Protein Assay Kit (Abcam, Cambridge, UK). Equal amounts of protein lysates mixed evenly with 6× loading buffer (5 : 1, V/V) were transferred to PVDF membranes. After blocking in 5% BSA for 2 h, the membranes were incubated with antibodies against p21 and p27 (1 : 1000, Cell Signaling Technology, Inc., Danvers, MA, USA), SM22ɑ, (1 : 1000, Abcam, Cambridge, UK), and mouse anti-rat/rab *β*-actin (1 : 1000, Cell Signaling Technology, Inc., Danvers, MA, USA) at 4°C overnight. Then, the membranes were incubated with HRP-conjugated secondary antibody at room temperature for 1 to 2 h, and chemiluminescent autography was performed using an ECL kit (Beyotime Biotechnology, Beijing, China). The grey values of the protein bands were analysed using the image processing software Image-Lab version 5.0 (Bio-Rad; Hercules, CA, USA).

### 2.11. Luciferase Assay

To verify miR-128-5p targeting of the p21 gene, wild-type (wt) and mutant-type (mut) 3′UTR sequence binding sites of the p21 gene were cloned into PGL3-CMV-LUC-MCS vectors using XhoI and MluI restriction sites. HEK-293 cells were cotransfected with pRL-TK vectors, pGL3 vector control, miR-128-5p mimic, or mimic-negative controls by using Lipofectamine® 2000 (Invitrogen, CA, USA). After incubation for 48 h, firefly luciferase activity was detected using dual-luciferase assays (Genomeditech, Shanghai, China). The results were normalized to a Renilla luciferase expression control.

### 2.12. Statistical Analysis

The results are presented as the mean ± SD. Statistical analysis was performed using the statistical software SPSS version 21.0 and assessed by one-way analysis of variance (ANOVA) or two-tailed Student's t-test to compare two treatments. A *p* value < 0.05 was considered statistically significant.

## 3. Results

### 3.1. AA and U0126 Suppress the Migration of ox-LDL-Treated VSMCs

A wound-healing assay was used to evaluate the role of AA on VSMC migration. The control group had a small amount of VSMC migration, and ox-LDL (50 mg·L-1) treatment significantly promoted cell migration (^*∗*^*P* < 0.05, Figure 1). However, both AA and U0126 (10 *μ*mol·L-1) treatment remarkably suppressed the migration ability of ox-LDL-treated VSMCs (^#^*P* < 0.05, Figure 1).

### 3.2. AA and U0126 Elevate SM22*α* Expression in ox-LDL-Treated VSMCs

SM22*α* is a marker protein for the contractile phenotype. Immunofluorescence assays revealed that ox-LDL treatment reduced the mean optical density of SM22*α* expression (^*∗∗*^*P* < 0.01, Figure 2). Treatment with AA and U0126 caused elevation of SM22*α* expression in ox-LDL-induced VSMCs (^#^*P* < 0.05, ^##^*P* < 0.01, Figure 2), indicating that AA and U0126 treatment could inhibit the conversion of VSMCs from a contractile to a synthetic phenotype induced by ox-LDL.

### 3.3. AA and U0126 suppress ox-LDL-induced MMP-2 and MMP-9 Secretion in VSMCs

MMP-2 and MMP-9 have been shown to be involved in cell migration and proliferation. ELISA was used to detect the expression of MMP-9 and MMP-2 in the supernatant of the cell culture. ox-LDL treatment significantly induced the expression of MMP-2 and MMP-9 compared with the control group (^*∗∗*^*P* < 0.01, Figure 3). However, treatment with AA and U0126 significantly repressed MMP-2 and MMP-9 expression in ox-LDL-treated VSMCs (^#^*P* < 0.05, ^##^*P* < 0.01, Figure 3).

### 3.4. AA and U0126 Inhibit ox-LDL-Induced VSMC Proliferation

Flow cytometry indicated that ox-LDL increased the number of BrdU-positive cells (new proliferation of VSMCs) (^*∗*^*P* < 0.05, Figure 4), while AA and U0126 treatment decreased the number of BrdU-positive VSMCs, at 24 h (^#^*P* < 0.05, ^##^*P* < 0.01, Figure 4), showing that AA and U0126 could inhibit the proliferation of cells.

### 3.5. AA and U0126 Regulate MicroRNA Expression in ox-LDL-Treated VSMCs

To further examine the effects of miRNAs on ox-LDL-induced VSMC treatment with AA or U0126, miRNA microarray analysis was applied to test miRNA expression in VSMCs induced by ox-LDL. miRNA microarray assays demonstrated that various miRNA expression levels among groups and ox-LDL treatment upregulated 7 miRNAs and downregulated 4 miRNAs in VSMCs compared to the control group (*P* < 0.01, Figures 5(a) and 5(b)). AA dramatically inhibited the overexpression of 6 miRNAs and upregulated 10 miRNAs in ox-LDL-treated VSMCs (*P* < 0.01, Figures 5(a) and 5(b)). ERK1/2 blocker U0126 treatment upregulated 9 miRNAs and downregulated 25 miRNAs in ox-LDL-treated VSMCs (*P* < 0.01, Figures 5(a) and 5(b)). Furthermore, we found that ox-LDL downregulated the expression of miR-466f-3p and miR-425-3p, while AA and U0126 treatment reversed this effect (Table 1). The overexpression of miR-27a-5p and miR-128-5p in ox-LDL-treated VSMCs was dramatically inhibited by treatment with AA and U0126 (Figures 5(a) and 5(b), Table 1). The sequences of miRNAs are shown in Table 2. Target genes of miRNAs were analysed according to the TargetScan 7.2 database and miRDB. Both miR-466f-3p and miR-425-3p negatively regulate cyclins, cyclin-dependent kinases (CDKs), and MMPs. Peroxisome proliferator-activated receptor (PPAR)ɑ, PPAR*δ*, p21, silent information regulator 2 (SIRT2), TIMP4, and TIMP3 are the target genes of miR-128-5p and miR-27a-5p, indicating that AA could alter miRNA expression in ox-LDL-induced VSMCs and regulate the expression of MMPs-TIMPs, p21-cyclins, and ERK1/2 inhibitor, which is related to the migration, phenotypic transformation, and proliferation of VSMCs (Figure 5(c)).

### 3.6. miR-128-5p Promotes the Migration, Phenotypic Transformation, and Proliferation of VSMCs

Because miR-128-5p negatively regulates p21, PPAR, SIRT2, and TIMP expression, we assumed that miR-128-5p could influence the migration, phenotypic transformation, and proliferation of VSMCs. We transfected the miR-128-5p mimic and inhibitor to test the role of miR-128-5p in the biological behaviours of VSMCs. The level of miR-128-5p expression was detected by qRT–PCR. The miR-128-5p mimic promoted the expression of miR-128-5p (^*∗*^*P* < 0.05), and the miR-128-5p inhibitor suppressed the levels of miR-128-5p (^#^*P* < 0.05) (Figure 6(a)). Scratch wound-healing assays showed that the miR-128-5p mimic promoted the migration of VSMCs (^*∗*^*P* < 0.05, Figure 6(b)), and the inhibitor reduced the migration rate of VSMCs compared with the NC groups (^#^*P* < 0.05, Figure 6(b)). Immunofluorescence assays and WB were applied to detect SM22*α* expression in VSMCs. The mimic suppressed SM22*α* expression (^*∗*^*P* < 0.05, Figure 7) and the inhibitor elevated SM22*α* fluorescent expression in VSMCs (^#^*P* < 0.05, Figure 7) compared with the NC groups. The same results were confirmed by WB: the mimic inhibited SM22ɑ expression (^*∗*^*P* < 0.055, Figure 8(a)), and the inhibitor increased SM22ɑ expression (^#^*P* < 0.05, Figure 8(a)), suggesting that miR-128-5p overexpression could induce VSMC transformation from a contractile to a synthetic phenotype.

The effect of miR-128-5p on the proliferation of VSMCs was detected by WB and immunocytochemistry staining of incorporated BrdU. The results showed that the miR-128-5p mimic suppressed p21 and p27 expression and that the inhibitor increased p21 and p27 expression compared to that in the NC (^*∗*^*P* < 0.05, ^#^*P* < 0.05, respectively, Figure 8(a)). This finding suggests that miR-128-5p can influence the cell cycle and affect VSMC proliferation. Immunocytochemistry staining of BrdU showed that the miR-128-5p mimic increased the number of proliferating VSMCs and the inhibitor repressed the proliferation of VSMCs compared to those in the NC groups (^*∗*^*P* < 0.05, ^#^*P* < 0.05, respectively, Figure 8(b)). The overexpression of miR-128-5p induced the proliferation of VSMCs, while the inhibitor reversed the results. Furthermore, both AA and U0126 treatment reduced the proliferation of VSMCs induced by mimic transfection compared with that in the mimic group (Δ*P* < 0.05, Figure 8(b)), suggesting that inhibition of the miRNAs could be a promising therapy for VSMC proliferation and that AA suppressed VSMC proliferation by repressing miR-128-5p expression as well as ERK1/2 inhibitor.

### 3.7. P21 Is the Direct Target of miR-128-5p

Based on TargetScan (http://www.targetscan.org/vert_71/) and miRDB (http://mirdb.org/), the p21 gene is a potential target of miR-128-5p (Figure 9(a)). To explore the role of miR-128-5p in the regulation of p21 expression, HEK-293 cells were cotransfected with a Renilla luciferase reporter vector containing the wild-type (wt) p21 3′UTR and mutant (mut) p21 3′UTR, UTR NC, and mimic NC. Our results showed that firefly luciferase activity in p21 3′UTR (wt)-transfected cells was lower than that in control cells (^*∗*^*P* < 0.05, Figure 9(b)). However, there was less effect of miR-128-5p on the luciferase activity in cells containing mutant p21 3′UTR (mut) (Figure 9(b)). Our results demonstrate that miR-128-5p directly binds to the 3′UTR sequence sites of the p21 gene.

## 4. Discussion

As an ancient classical traditional Chinese medicinal formula, the compatibility of Alisma orientalis and Atractylodes macrocephala was first described in the Eastern Han Dynasty and exhibited a wide range of bioactivities in diverse cells [9, 19–23]. Until now, its effect on the migration, phenotypic transformation, and proliferation of VSMCs induced by ox-LDL remained unclear.

Several studies have reported that phenotypic transformation of VSMCs is a crucial process and promotes VSMC proliferation and migration in the process of AS5. Our study verified that the migration, phenotypic transformation, and proliferation abilities of ox-LDL-treated VSMCs were higher than those of control VSMCs. Previous studies demonstrated that AA could inhibit the phosphorylation of ERK1/29, and AA suppressed the migration, transformation, and proliferation abilities of ox-LDL-treated VSMCs as well as ERK1/2 blockers in the present study, suggesting that AA could affect the biological behaviours of VSMCs, which is associated with the inhibition of the ERK1/2 signalling pathway.

miRNAs are conserved, small and single-stranded noncoding RNAs that negatively regulate gene expression at the posttranscriptional level and therefore, repress protein expression. Accumulating evidence reveals that miRNAs serve as important regulators of a range of behaviours of VSMCs and are involved in molecular signalling pathways of AS10-12. In the present study, ox-LDL induced overexpression of miR-27a-5p and miR-128-5p and downregulated miR-466f-3p and miR-425-3p expression. AA and U0126 inhibited the expression of miR-27a-5p and miR-128-5p and elevated miR-466f-3p and miR-425-3p expression in ox-LDL-induced VSMCs. A previous study showed that the main active ingredient of AA-inhibited ERK1/2 phosphorylation9, suggesting that AA could inhibit ox-LDL-induced VSMC migration, transformation, and proliferation by regulating the expression of these miRNAs, which could be associated with the ERK1/2 pathway.

Cyclins are recognized as important mediators in the cell cycle [24]. As negative regulators of cyclins, p27 and p21 exert a central role in cell cycle arrest [25, 26]. The activity of cyclin-dependent kinases (CDKs) is strongly linked to the expression of cyclins, which can initiate DNA synthesis, promote the cell cycle, and play an important role in cell proliferation [27–29]. P21 prevents DNA replication from inhibiting cell proliferation through the control of CDK2, CDK4, and CDK6. Cyclins and CDKs are the target genes of miR-466f-3p and miR-425-3p, and p21 is the target gene of miR-128-5p according to the TargetScan7.1 database. Our study showed that miR-128-5p directly targeted the 3′UTRs of the p21 gene, suppressed p21 expression and induced the proliferation of VSMCs. Inhibition of miR-128-5p increased the levels of p21 and p27 expression and then inhibited proliferation. AA and U0126 treatment suppressed the increasing number of VSMCs induced by miR-128-5p overexpression. Treatment with AA and ERK1/2 inhibitor effectively suppressed the proliferation of VSMCs by inhibiting miR-128-5p in ox-LDL-induced VSMCs, indicating that AA could inhibit VSMC proliferation by suppressing miR-128-5p expression, which is closely linked to the ERK1/2 signalling pathway.

TIMPs play a central role in suppressing the activation of MMPs. TIMPs and MMPs have been identified as key molecules in vascular remodeling and are linked to VSMC proliferation and migration [30–33]. SM22*α* is a contractile marker of VSMCs that affects the proliferation of VSMCs and the development of AS5. We detected that treatment with AA and U0126 effectively increased the expression of SM22*α* and suppressed the levels of MMP-2 and MMP-9 in VSMCs exposed to ox-LDL. It has been reported that several miRNAs contribute to an SMC-specific transcriptional program in regulating VSMC phenotypic transformation and proliferation [34]. In the present study, AA and U0126 obviously suppressed the expression of miR-27a-5p and miR-128-5p, and elevated miR-466f-3p and miR-425-3p expression in ox-LDL-treated VSMCs. MMP-11, MMP-13, and MMP-19 are negatively regulated by miR-466f-3p and miR-425-3p. TIMP-3, TIMP-4, PPARɑ, PPAR*δ*, and SIRT2 are the target genes of miR-27a-5p and miR-128-5p according to the TargetScan 7.1 database. Inhibition of SIRT2 represses the proliferation and synthetic phenotypic transformation of VSMCs [35]. Activation of PPAR*ɑ* and PPAR*γ* can attenuate VSMC proliferation and migration [36–38] and exert a protective effect on AS [39]. Furthermore, miR-27a and miR-128 suppress the LDL receptor and dysregulate cholesterol homeostasis, which is involved in cholesterol efflux and represses the progression of AS [40, 41]. Therefore, we assumed that AA could suppress VSMC migration, phenotypic transformation, and proliferation by altering the expression of these miRNAs and exert multiple roles in the process of AS.

It has been reported that overexpression of miR-128 can significantly decrease VSMC migration, phenotypic transformation, and proliferation by targeting Kruppel-like factor 4 (KLF4) [42]. KLF4 acts as a key repressor of VSMC differentiation, modulating the expression of SM22*α* and PPARs [42, 43]. miR-128-5p has a similar function as miR-128 and TIMP-3, and TIMP-4, SIRT2, PPARɑ, PPAR*δ*, and p21 are suppressed by miR-128-5p. We hypothesized that miR-128-5p could affect the migration, phenotypic transformation, and proliferation of VSMCs. The results showed that the miR-128-5p mimic increased the migration, phenotypic transformation, and proliferation of VSMCs. The inhibition of miR-128-5p elevated SM22*α* expression and suppressed the migration and proliferation of VSMCs, suggesting that inhibition of miR-128-5p may be a promising treatment for the progression of AS. AA and U0126 treatment reduced the increase in VSMC proliferation induced by miR-128-5p mimic transfection compared with that in the mimic group, indicating that AA and U0126 could inhibit VSMC proliferation by repressing miR-128-5p expression. The p21 protein is involved in cell proliferation, and the 3′UTR of the p21 gene contains the binding sequence sites of miR-128-5p. Luciferase assays showed that p21 was the direct target gene of miR-128-5p. The miR-128-5p mimic induced overexpression of miR-128-5p, blocked p21 expression, and increased VSMC proliferation. AA and ERK1/2 blockers suppressed VSMC proliferation by repressing miR-128-5p expression. This finding indicates that miR-128-5p can effectively inhibit the proliferation of VSMCs by targeting p21 expression and that AA alters the behaviours of VSMCs by arresting miR-128-5p expression by targeting the p21 gene.

## 5. Conclusion

In conclusion, the results of our study verify that treatment with AA and ERK1/2 blockers inhibits ox-LDL-stimulated VSMC migration, phenotypic transformation, and proliferation by regulating the expression of miR-466f-3p, miR-425-3p, miR-27a-5p, and miR-128-5p, especially by suppressing miR-128-5p and by targeting the p21 gene. This study provides new insights into how AA regulates the biological behaviours of VSMCs and exerts multiple roles in the process of AS.

## Figures and Tables

**Figure 1:** Effects of AA and U0126 on VSMC migration. VSMCs were pretreated with ox-LDL (50 mg·L-1), AA, and U0126 (10 *μ*mol·L-1) for 24 h three independent experiments were performed. The results are presented as the mean ± SD (*n* = 3). ^*∗*^*P* < 0.05 versus the control group; ^#^*P* < 0.05 versus the ox-LDL group.

**Figure 2:** Effects of AA and U0126 on the expression of SM22ɑ protein in VSMCs treated with ox-LDL. Data are representative of 3 experiments. Following treatment with ox-LDL (50 mg·L-1), AA, and U0126 (10 *μ*mol·L-1) for 24 h, SM22*α* expression was detected by immunofluorescence (*n* = 5). ^*∗∗*^*P* < 0.01 versus the control group; ^#^*P* < 0.05 and ^##^*P* < 0.01 versus the ox-LDL group.

**Figure 3:** AA and U0126 inhibit ox-LDL-induced upregulation of MMP-2 and MMP-9 in VSMCs. Six independent experiments were repeated. ELISA detected secreted MMP-9 and MMP-2 expression in the culture medium (*n* = 6). ^*∗∗*^*P* < 0.01 versus the control group; ^#^*P* < 0.05 and ^##^*P* < 0.01 versus the ox-LDL group.

**Figure 4:** AA and U0126 repress ox-LDL-induced VSMC proliferation. The numbers of BrdU-positive cells and total cells were calculated. These data are representative of 3 experiments. The results are described as the mean ± SD (*n* = 3). ^*∗*^*P* < 0.05 versus the control group; ^#^*P* < 0.05 and ^##^*P* < 0.01versus the ox-LDL group.

**Figure 5:** AA and U0126 regulate microRNA expression in ox-LDL-treated VSMCs. (a) miR-466f-3p, miR-425-3p, miR-27a-5p, and miR-128-5p were significantly associated with AA and U0126 treatment in ox-LDL-treated VSMCs (*P* < 0.01). (b) miRNA microarray assays show that AA and U0126 regulate the expression of various miRNAs in ox-LDL-treated VSMCs. (c) According to the TargetScan 7.1 database and miRDB, PPARs, p21, SIRT2, and TIMPs are potential targets of miR-128-5p and miR-27a-5p, and cyclins, CDKs, and MMPs are the potential targets of miR-466f-3p and miR-425-3p.

**Figure 6:** Transfection of VSMCs with miR-128-5p mimic and inhibitor. (a) The expression of miR-128-5p was detected by qRT–PCR. These data are representative of 6 experiments. The results are described as the mean ± SD (*n* = 6). ^*∗*^*P* < 0.05 versus mimic NC and ^#^*P* < 0.05 versus inhibitor NC. (b) The migration of VSMCs was detected after transfection. These data are representative of 6 experiments. The results are described as the mean ± SD (*n* = 6). ^*∗*^*P* < 0.05 versus mimic NC and ^#^*P* < 0.05 versus inhibitor NC.

**Figure 7:** Transfection of miR-128-5p affects phenotypic transformation. SM22ɑ expression was detected by immunofluorescence assay. These data are representative of 3 experiments. The results are described as the mean ± SD (*n* = 3). ^*∗*^*P* < 0.05 versus mimic NC and ^#^*P* < 0.05 versus inhibitor NC.

**Figure 8:** Transfection of the miR-128-5p mimic and inhibitor affected SM22ɑ, p21 and p27 expression, and VSMC proliferation. (a) Western blotting was performed to determine the expression of sm22ɑ, p21, and p27. These data are representative of 3 experiments. The results are described as the mean ± SD (*n* = 3). ^*∗*^*P* < 0.05 versus mimic NC and ^#^*P* < 0.05 versus inhibitor NC. (b) Immunocytochemistry staining of incorporated BrdU in VSMCs was performed to investigate the proliferation of VSMCs. These data are representative of 3 experiments. The results are described as the mean ± SD (*n* = 3). ^*∗*^*P* < 0.05 versus mimic NC, ^#^*P* < 0.05 versus inhibitor NC, and Δ*P* < 0.05 versus mimic NC.

**Figure 9:** The p21 gene is the direct target of miR-128-5p. (a) The predicted miR-128-5p binding sequences in the p21 gene and the designed mut sequence (p21-mut). (b) The miR-128-5p mimic was cotransfected with the wild-type or mutated p21 3′UTR sequence vectors in HEK 293T cells. The relative firefly luciferase activity was calculated. Three independent experiments were repeated. ^*∗*^*P* < 0.05 versus the respective NC.

**Table 1:** Expression of individual miRNAs.

miRNAs	Control	ox-LDL	AA	U0126
miR-128-5p	45.27 ± 8.74	73.68 ± 8.77^##^	48.41 ± 10.39^∗∗^	39.75 ± 6.71^@@^
miR-27a-5p	907.26 ± 35.52	1,091.40 ± 96.31^##^	736.02 ± 10.19^∗∗^	568.15 ± 82.00^@@^
miR-425-3p	276.48 ± 19.89	198.52 ± 24.70^##^	244.03 ± 15.00^*∗*^	259.94 ± 20.42^@^
miR-466f-3p	58.26 ± 3.31	25.34 ± 1.31^##^	41.94 ± 6.19^∗∗^	34.06 ± 1.33^@^

^#^ *P* < 0.05, ^##^*P* < 0.01 versus control; ^*∗*^*P* < 0.05, ^*∗∗*^*P* < 0.01 versus ox-LDL, ^@^*P* < 0.05, ^@@^*P* < 0.01 versus ox-LDL.

**Table 2:** The sequences of individual members in miRNAs.

miRNAs	Sequences
miR-128-5p	CGGGGCCGTAGCACTGTCTGAGA
miR-27a-5p	AGGGCTTAGCTGCTTGTGAGCA
miR-425-3p	CATCGGGAATATCGTGTCCGCC
miR-466f-3p	TACACACACACATACACACAGA

## Data Availability

The data that support the findings of this study are available from the corresponding author upon reasonable request.
